# Effect of Amoxicillin and Clavulanate Potassium Combined with Bazhengsan on Pediatric Urinary Tract Infection

**DOI:** 10.1155/2021/4575503

**Published:** 2021-10-20

**Authors:** Shengjun Zhang, Zhenghua Wang, Guoping Xu

**Affiliations:** ^1^Department of Pediatric Surgery, People's Hospital of Rizhao, Rizhao 276826, Shandong Province, China; ^2^Department of Surgery, Rizhao Maternal and Child Health Care Hospital, Rizhao 276800, Shandong Province, China; ^3^Department of Urology and Anorectology, Wuhan Xinzhou District People's Hospital, Wuhan 430400, Hubei Province, China

## Abstract

**Objective:**

To explore the therapeutic effect of amoxicillin and clavulanate potassium combined with Bazhengsan on pediatric urinary tract infection (UTI).

**Methods:**

The data of 120 UTI children treated in Wuhan Xinzhou District People's Hospital from February 2019 to February 2020 were retrospectively analyzed. They were equally split into experimental group (EG) and control group (CG) according to the order of admission. All children were treated with amoxicillin and clavulanate potassium for suspension (twice a day), and EG was additionally treated with one dose of Bazhengsan daily. Both groups were treated for 10 days. After treatment, the immune function indexes, inflammatory factor levels, and clinical efficacy were compared before and after treatment.

**Results:**

No remarkable differences in the general data such as blood routine and urine routine results were observed between the two groups before treatment (*P* > 0.05). After treatment, EG achieved obviously better immune function indexes (*P* < 0.001) and lower levels of inflammatory factors (*P* < 0.05) compared with CG. Besides, the treatment effective rate in EG (96.7%) was higher than that in CG (*P* < 0.05).

**Conclusion:**

Amoxicillin and clavulanate potassium combined with Bazhengsan can improve the immune function of UTI children and reduce the levels of inflammatory factors, with remarkable effects, which should be popularized in practice.

## 1. Introduction

Pediatric urinary tract infection (UTI) refers to urinary tract inflammation caused by pathogens invading urinary tract mucosa or tissue. Its clinical manifestations mainly include abnormal urination such as frequency and urgency of urination, as well as urinary incontinence and retention in some children [1, 2]. If not treated in time, it may trigger chronic urinary system infection and lead to renal fibrosis, seriously endangering children's physical and mental health. Antibiotics are the main treatment measures in clinic since UTI is mostly caused by bacteria. However, the wide application of antibiotics results in antibiotic resistance in more than half of the strains due to the production of *β*-lactamase [3, 4]. Therefore, children can be treated with *β*-lactamase inhibitors in practice to protect the activity of *β*-lactamase antibiotics. Amoxicillin and clavulanate potassium is a mixture of the *β*-lactam antibiotic (amoxicillin) with the *β*-lactamase inhibitor (clavulanate potassium), which can enhance the sensitivity of pathogens to amoxicillin and inhibit the production of drug-resistance bacteria [5]. At present, many reports have shown that amoxicillin and clavulanate potassium can reduce the clinical symptoms of UTI children, and especially oral administration of this drug can reduce the incidence of complications such as phlebitis, with definite efficacy [6, 7]. However, UTI can recur in children due to factors such as immunocompromise, and recurrence is an important reason for the development of UTI into chronic renal failure [8, 9]. However, amoxicillin and clavulanate potassium cannot improve the immune function of children, so it is extremely important to combine it with other therapeutic drugs.

In recent years, traditional Chinese medicine (TCM) with the holistic view has shown unique advantages in the treatment of urinary tract diseases. TCM classifies UTI into the category of stranguria and holds that the disease in children is caused by excessive milk and food and accumulation of heat and stagnation, which triggers disturbance of qi transformation and urinary tract obstruction, resulting in frequent urination and pain [10, 11]. The treatment should be based on clearing heat, eliminating accumulation, promoting urination, and removing stranguria. Ning treated pediatric UTI with Bazhengsan and found that *Polygonum aviculare* and fringed pink in the medicine inhibited *Staphylococcus* and *Bacillus* and turned bacteriuria negative [12]. In addition, scholars Changli Xue found that the total effective rate (98.3%) of children was significantly improved compared with the control group after the addition and subtraction treatment of Bazhengsan, suggesting the remarkable effects of this drug on UTI [13]. However, the research of Bazhengsan in UTI treatment focuses on the short-term efficacy, and its impact on immune function and inflammatory factor levels in children remains unclear. Besides, there is no study on the application of Bazhengsan combined with amoxicillin and clavulanate potassium. Based on this, this paper will explore the actual effect of the combined treatment on pediatric UTI, reported as follows.

## 2. Materials and Methods

### 2.1. Study Design

This retrospective study was conducted in Wuhan Xinzhou District People's Hospital from February 2019 to February 2020, aiming to explore the efficacy of amoxicillin and clavulanate potassium combined with Bazhengsan in the treatment of pediatric UTI.

### 2.2. Recruitment of Research Subjects

The data of UTI children treated in Wuhan Xinzhou District People's Hospital from February 2019 to February 2020 were retrospectively analyzed. Children meeting the following criteria were included: (1) children who were diagnosed with UTI by examination, meeting the criteria of Guidelines for the Clinical Research of Chinese Medicine New Drugs [14] and Zhu Futang Practical Pediatrics (7th Edition) [15], that is, white blood cell (WBC) in urine routine >5/HP, and midstream urine culture colony count >1 × 10^6^/mL; (2) children with typical urinary tract irritation symptoms; (3) children who were treated throughout the whole period in our hospital without transferring or stopping treatment; (4) children with complete clinical; and (5) children between 1–12 years old. Children were excluded according to the following criteria: (1) children with urinary calculi, urinary deformity, deformity of kidney, chronic pyelonephritis, or other serious organic diseases; (2) children quitting the treatment halfway and changing the treatment plans; (3) children with simple urethral syndrome; (4) children who were allergic to the drugs involved in the study; (5) children with missing clinical data; and (6) children who received antibacterial drug therapy before participating in the study.

### 2.3. Steps

A total of 120 children were enrolled in this study and were equally split into experimental group (EG) and control group (CG) according to the order of admission. On the day when the family members agreed to participate in the study, the research group collected social demographic data and clinical data of the children and tested their blood routine, urine routine, immune function, and inflammatory factor levels. At 10 days after treatment, the research group tested their immune function and inflammatory factor levels again.

### 2.4. Ethical Considerations

This study is in line with the principles of Declaration of Helsinki (as revised in 2013) [16] and approved by the ethics committee of Wuhan Xinzhou District People's Hospital. After the children were recruited, the research group explained the purpose, significance, content, and confidentiality of the study to their families and asked them to sign the informed consent.

### 2.5. Withdrawal Criteria

Judged by the research group, the children with the following conditions were unsuitable to continuously participate in the experiment, and their medical records would be kept but not for data analysis: (1) adverse events or serious adverse events occurred; (2) the condition deteriorated during the experiment; (3) the subjects had some serious comorbidities or complications; and (4) the families of the children were unwilling to continue the clinical trial and requested the research group for withdrawal.

### 2.6. Methods

All children took amoxicillin and clavulanate potassium for suspension (Guangzhou Baiyunshan Pharmaceutical Co., Ltd., Baiyunshan Pharmaceutical General Factory, National Medical Products Administration approval no. H20041109, each containing 200 mg of amoxicillin and 28.5 mg of clavulanate with the ratio as 7 : 1), with the specific administration methods as follows: (1) 14.3 mg/kg each time for children with the body weight less than 13 kg and age less than 2 years old; (2) one pack each time for children with the body weight of 13–21 kg; and (3) 2 packs each time for those with body weight over 21 kg. After the symptoms disappeared, children continued to take the suspension orally. The total treatment time was 10 days.

EG was additionally treated with Bazhengsan consisting of plantain seed, *Polygonum aviculare*, fringed pink, talc, ural licorice root tip, *Gardenia*, rhubarb, dandelion, and *Hedyotis diffusa*. With the addition and subtraction of herbs in Bazhengsan, Cortex Phellodendri and *Bupleurum* were added for children with fever and chills, Lalang Grass Rhizome and field thistle were added for children with hematuria, peony and *Cyperus rotundus* were added for children with abdominal distention, and *Astragalus mongholicus* and *Codonopsis* were added for those with qi deficiency. Bazhengsan was decocted by the research group and administrated specifically as follows: (1) 1 dose every 2 days with frequent administration every day for children aged under 2 years old; (2) 1 dose every 2 days and three times a day for children aged 2–5 years old; and (3) 1 dose every day and three times a day for children over 5 years old. The total treatment time was 10 days.

### 2.7. Observation Criteria

#### 2.7.1. General Data

The general data extraction forms were established by the children's families, including inpatient number, name, gender, age, urine culture results, blood routine results, urine routine results, residence, family monthly income, parents' marital status, and parents' educational level.

#### 2.7.2. Immune Function Indexes

Five milliliter of fasting venous blood was taken from children before treatment (T_1_), 5 days after treatment (T_2_), and 10 days after treatment (T_3_). The levels of T lymphocyte subsets (CD8^+^ and CD4^+^/CD8^+^) were detected by flow cytometry (ACEA BIO Hangzhou Co., Ltd, Zhejiang Medical Products certified no. 20142400581), and the levels of immunoglobulin (IgA and IgG) were measured by nephelometry immunoassay kit (Nanjing Getein Bio-Pharmaceutical Co., Ltd., Jiangsu Medical Products certified no. 20122400146).

#### 2.7.3. Inflammatory Factor Levels

Five milliliter of fasting venous blood was collected at T_1_, T_2_, and T_3_. The levels of tumor necrosis factor-*α* (TNF-*α*), interleukin-6 (IL-6), high-sensitivity C-reactive protein (hs-CRP), and procalcitonin (PCT) were measured by enzyme-linked immunosorbent assay (Beijing Kewei Clinical Diagnostic Reagent Inc., National Medical Products Administration approval no. S20060028).

#### 2.7.4. Clinical Efficacy

The therapeutic efficacy of the children was evaluated according to the Guidelines for Clinical Research on Antibiotics [17] issued by the Pharmaceutical Administration of the Ministry of Health. If the symptoms, signs, laboratory tests, and etiological tests were normal, the children were regarded as cured; if the condition of the children was remarkably improved while one index did not return to a normal level, the treatment was deemed as markedly effective; if the condition was improved while more than one index did not return to normal levels, the treatment was classified as effective; if the condition was not improved, or even aggravated, the treatment was ineffective.

### 2.8. Statistical Processing

The data in this study were processed by SPSS20.0 software and graphed by GraphPad Prism 7 (GraphPad Software, San Diego, USA). The data included in the study were enumeration data (clinical efficacy) and measurement data (immune function indexes and inflammatory factor levels), tested by *X*^2^ and *t*-test. The differences were statistically significant at *P* < 0.05.

## 3. Results

### 3.1. Comparison of General Data of Children

No remarkable differences in the general data such as blood routine and urine routine results were observed between the two groups before treatment (*P* > 0.05) (see Table 1).

### 3.2. Comparison of Immune Function Indexes of Children

The immune function indexes were obviously better in EG than in CG (*P* < 0.001) (see Figure 1).

Figure 1(a) shows IgA. With no remarkable difference in the IgA at T_1_ between the two groups (0.48 ± 0.05 vs 0.49 ± 0.04, *P* > 0.05), the IgA at T_2_ and T_3_ was obviously higher in EG than in CG (0.70 ± 0.09 vs 0.53 ± 0.06, 0.85 ± 0.07 vs 0.69 ± 0.04, *P* < 0.001).

Figure 1(b) shows IgG. With no remarkable difference in the IgG at T_1_ between the two groups (5.41 ± 0.54 vs 5.43 ± 0.56, *P* > 0.05), the IgG at T_2_ and T_3_ was obviously higher in EG than in CG (7.23 ± 0.75 vs 6.21 ± 0.60, 8.67 ± 0.85 vs 6.54 ± 0.65, *P* < 0.001).

Figure 1(c) shows CD8^+^. With no remarkable difference in the CD8^+^ at T_1_ between the two groups (32.98 ± 3.21 vs 32.96 ± 3.24, *P* > 0.05), the CD8^+^ at T_2_ and T_3_ was obviously lower in EG than in CG (27.41 ± 2.54 vs 30.58 ± 2.45, 23.12 ± 1.22 vs 25.87 ± 1.35, *P* < 0.001).

Figure 1(d) shows CD4^+^/CD8^+^. With no remarkable difference in the CD4^+^/CD8^+^ at T_1_ between the two groups (1.12 ± 0.12 vs 1.14 ± 0.13, *P* > 0.05), the CD4^+^/CD8^+^ at T_2_ and T_3_ was obviously higher in EG than in CG (1.42 ± 0.23 vs 1.21 ± 0.20, 1.64 ± 0.36 vs 1.32 ± 0.35, *P* < 0.001).

### 3.3. Comparison of Inflammatory Factors in Children

The levels of inflammatory factors in EG were significantly lower than those in CG (*P* < 0.001) (see Figure 2).

Figure 2(a) shows TNF-*α*. With no remarkable difference in the TNF-*α* at T_1_ between the two groups (125.65 ± 12.10 vs 125.84 ± 12.41, *P* > 0.05), the TNF-*α* at T_2_ and T_3_ was obviously lower in EG than in CG (109.98 ± 10.14 vs 118.64 ± 12.65, 101.98 ± 9.65 vs 116.98 ± 11.41, *P* < 0.001).

Figure 2(b) shows IL-6. With no remarkable difference in the IL-6 at T_1_ between the two groups (154.52 ± 12.98 vs 154.60 ± 12.48, *P* > 0.05), the IL-6 at T_2_ and T_3_ was obviously lower in EG than in CG (100.65 ± 10.22 vs 115.98 ± 11.50, 50.98 ± 6.98 vs 70.41 ± 7.68, *P* < 0.001).

Figure 2(c) shows hs-CRP. With no remarkable difference in the hs-CRP at T_1_ between the two groups (6.54 ± 0.68 vs 6.55 ± 0.67, *P* > 0.05), the hs-CRP at T_2_ and T_3_ was obviously lower in EG than in CG (4.26 ± 0.54 vs 5.31 ± 0.58, 3.10 ± 0.35 vs 4.22 ± 0.36, *P* < 0.001).

Figure 2(d) shows PCT. With no remarkable difference in the PCT at T_1_ between the two groups (154.44 ± 21.68 vs 154.56 ± 21.54, *P* > 0.05), the PCT at T_2_ and T_3_ was obviously lower in EG than in CG (121.98 ± 12.21 vs 134.85 ± 12.68, 104.98 ± 10.68 vs 115.68 ± 11.45, *P* < 0.001).

### 3.4. Comparison of Clinical Efficacy in Children

The clinical efficacy in EG was remarkably better compared with CG (*P* < 0.05) (see Table 2).

## 4. Discussion

The incidence of pediatric urinary tract infection (UTI) is 3%–5% in China [18], and the children present with different symptoms and signs due to different ages and urinary infection sites. Gram-negative bacteria are the most common pathogens, and the proportion of Gram-positive bacteria represented by *Streptococcus faecalis* and *Staphylococcus* has also increased in recent years. Antibiotics are still the main treatment measures. Antibiotics are secondary metabolites with antipathogen effects, which can selectively act on specific links in the synthesis of deoxyribonucleic acid and ribonucleic acid with protein in bacterial cells, so as to inhibit, kill, and dissolve bacteria. Early antibiotic treatment of pediatric UTI has achieved remarkable results. However, with the long-term administration of antibiotics, the drug-resistant bacteria have secreted a large amount of *β*-lactamase against *β*-lactam antibiotics, which can cleave the *β*-lactam ring, lose the antibacterial activity, and subsequently enhance the bacterial resistance to antibiotics such as penicillin and cephalosporin. In order to stabilize the antibacterial efficacy of antibiotics, children can be clinically treated with *β*-lactamase inhibitors that can irreversibly combine with *β*-lactamase to ensure the role of antibiotics [19]. Amoxicillin and clavulanate potassium are a mixture of the *β*-lactam antibiotic (amoxicillin) with the *β*-lactamase inhibitor (clavulanate potassium), in which the former has an antibacterial effect on Gram-negative and Gram-positive bacteria, while the latter has strong broad-spectrum enzyme inhibitory function. Their combination can enhance the sensitivity of antibiotics and reduce the possibility of drug-resistant bacteria. It has been well documented that amoxicillin and clavulanate potassium can alleviate the clinical symptoms of UTI children and improve the short-term efficacy [20], but it cannot reduce the recurrence rate of pediatric UTI. About 50% of children will relapse after 1 month of treatment due to complex factors, and kidney scars can be formed in severe cases, triggering secondary hypertension and chronic renal failure [21], with poor prognosis.

There are many reasons for the recurrence of pediatric UTI, and low immune function is one of the most critical factors. Once the immune balance is damaged, normal bacteria can become opportunistic pathogens, triggering the recurrence of UTI. Carmen and Maria and have shown in their study that the levels of T lymphocyte subsets in patients with chronic UTI are markedly lower than those in healthy people. They also have stated that the imbalance of CD4^+^/CD8^+^ is an important factor leading to immune disorders, and immunoglobulin also plays an important role in resisting bacterial invasion [22]. Bazhengsan in this study is derived from an ancient prescription, including plantain seed, *Polygonum aviculare*, fringed pink, talc, ural licorice root tip, *Gardenia*, rhubarb, dandelion, and *Hedyotis diffusa*. Plantain seed promotes urination, removes stranguria, clears heat, and brightens the eye because its outer epidermal cell wall contains a large number of hydrophilic polysaccharide colloids that can improve the intensity of delayed allergic reaction and increase the level of hemolysin in mice with low immune function, indicating that the substance can enhance the immune function. In addition to plantain seed, water extract and low polarity extract can also regulate the secretion of human immunoglobulin, while rhubarb can enhance the IgA level secreted by the intestinal tract of burned mice and accelerate the secretion of immune-related substances [23]. Therefore, Bazhengsan has an immune enhancement effect, and the immune function indexes of EG after treatment were significantly better compared with CG (*P* < 0.001).

At present, scholars have studied the application of Bazhengsan in pediatric UTI, but the effect of the drug on the levels of inflammatory factors in children remains unclear. *Polygonum aviculare* in Bazhengsan significantly inhibits *Shigella flexneri*, *Escherichia coli*, *Staphylococcus aureus*, and *Staphylococcus*, while the water and ethanol extracts of fringed pink also restrain *Escherichia coli* and *Salmonella paratyphi*. Moreover, dandelion and *Hedyotis diffusa* have strong inhibitory effects on a variety of bacteria and cocci, while rhubarb can also hinder the nucleic acid synthesis of bacterial cells and plays an anti-anaerobic role. Cao et al. have shown in their study that rhubarb can improve serum TNF-*α* and IL-6 levels, indicating that the drug can effectively prevent the amplification of inflammatory mediators and avoid their biological effects [24]. Therefore, the levels of inflammatory factors after treatment in this study were lower in EG than in CG (*P* < 0.001), with markedly better clinical efficacy in EG (*P* < 0.05).

It is worth noting that some scholars have found that rhubarb can inhibit the expression of intercellular attachment molecules in glomerulus, reduce the proliferation of human renal fibroblasts induced by mitogen PMA, and hinder the secretion of IL-6, thereby preventing renal fibrosis [25] or protecting the renal function of UTI children. This study did not discuss the renal function of children, and the protective effect of Bazhengsan on renal function of UTI children needs to be further explored.

In addition, amoxicillin and clavulanate potassium combined with Bazhengsan can enhance the comprehensive efficacy of children, which should be popularized in practice.

## Figures and Tables

**Figure 1:** Comparison of immune function indexes of children ($\bar{x}\pm s$). Note: the abscissa from left to right was T_1_, T_2_, and T_3_. The lines with dots were EG while those with squares were CG. # indicated *P* < 0.001.

**Figure 2:** Comparison of inflammatory factors in children ($\bar{x}\pm s$). Note: the abscissa from left to right was T_1_, T_2_, and T_3_. The black area was EG and the gray area was CG. # indicated *P* < 0.001.

**Table 1:** Comparison of general data of children.

Group	EG (*n* = 60)	CG (*n* = 60)	*X* ^2^/*t*	*P*
Gender			0.035	0.853
Male	25	24		
Female	35	36		
Age (years)				
Range	1–10	1–11		
Average age	6.54 ± 1.22	6.59 ± 1.20	0.226	0.821
Urine culture			—	—
Positive	60	60		
Negative	0	0		
Blood routine			0.100	0.752
WBC ≤ (11 × 10^9^)·L^−1^	54	55		
WBC > (11 × 10^9^)·L^−1^	6	5		
Urine routine			0.054	0.817
WBC > 20/HP	48	49		
5/HP < WBC < 19/HP	12	11		
Arterial blood gas indexes (mmHg)				
Residence			0.035	0.852
Urban area	36	37		
Rural area	24	23		
Family monthly income(yuan)			0.034	0.853
≥5000	35	34		
<5000	25	26		
Marital status of parents			0.152	0.697
Married	56	57		
Single/divorced/widowed	4	3		
Education level of parents			0.141	0.707
High school and below	24	22		
University and above	36	38		

**Table 2:** Comparison of clinical efficacy in children (*n*(%)).

Group	*N*	Cured	Markedly effective	Improved	Ineffective	Total effective rate
EG	60	30 (50.0)	18 (30.0)	10 (16.7)	2 (3.3)	58 (96.7)
CG	60	24 (40.0)	10 (16.7)	16 (26.7)	10 (16.7)	50 (83.3)
*X* ^2^		1.212	2.981	1.768	5.926	5.926
*P*		0.271	0.084	0.184	0.015	0.015

## Data Availability

The data used to support the findings of this study are available upon reasonable request from the corresponding author.
